The article "The Relationship between Serum Insulin-Like Growth Factor I Levels and Ischemic Stroke Risk" was retracted in 2022. Reasons: duplicate publication; signs of a paper mill; original data or images not available; concerns about the data.

# The Relationship between Serum Insulin-Like Growth Factor I Levels and Ischemic Stroke Risk

**DOI:** 10.1371/journal.pone.0094845

**Published:** 2014-04-11

**Authors:** Xiang Dong, Geng Chang, Xiao-Fei Ji, Ding-Bo Tao, Ying-Xin Wang

**Affiliations:** Department of Neurology, The First Affiliated Hospital of Dalian Medical University, Dalian, Liaoning Province, P.R. China; University of Warwick – Medical School, United Kingdom

## Abstract

**Objective:**

The aim of the study was to assess the relationship between insulin-like growth factor I (IGF-I) serum levels and acute ischemic stroke (AIS) in a Chinese population.

**Methods:**

All consecutive patients with first-ever AIS from August 1, 2011 to July 31, 2013 were recruited to participate in the study. The control group comprised 200 subjects matched for age, gender, and conventional vascular risk factors. IGF-I serum levels were determined by chemiluminescence immunoassay. The National Institutes of Health Stroke Scale (NIHSS) score was assessed on admission blinded to serum IGF-I levels.

**Results:**

The median serum IGF-1 levels were significantly (P = 0.011) lower in AIS patients (129; IQR, 109–153 ng/mL) compared with control cases (140; IQR, 125–159 ng/mL). We found that an increased risk of AIS was associated with IGF-I levels ≤135 ng/mL (unadjusted OR: 4.17; 95% CI: 2.52–6.89; P = 0.000). This relationship was confirmed in the dose-response model. In multivariate analysis, there was still an increased risk of AIS associated with IGF-I levels ≤135 ng/mL (OR: 2.16; 95% CI:1.33–3.52; P = 0.002) after adjusting for possible confounders.

**Conclusion:**

Lower IGF-I levels are significantly related to risk of stroke, independent from other traditional and emerging risk factors, suggesting that they may play a role in the pathogenesis of AIS. Thus, strokes were more likely to occur in patients with low serum IGF-I levels in the Chinese population; further, post-ischemic IGF-I therapy may be beneficial for stroke.

## Introduction

As the most common cause of neurologic disability, ischemic stroke is often associated with sensor motor and cognitive impairments due to neuronal degeneration. It causes a great financial burden because one third of surviving stroke patients remains dependent in daily activities.

Insulin-like growth factor I (IGF-I) is a single-chain polypeptide (70 amino acids) that shares homology with proinsulin [1]. Metabolic functions, particularly glucose metabolism, constitute an important aspect of IGF-I activities. The actions of IGFs are mediated by specific membrane receptors. The IGF system is composed of multiple receptors and ligands. It includes three ligands (IGF-I, IGF-II, and insulin), four receptors, at least six high-affinity binding proteins and binding protein proteases. IGF-I promotes macrophage chemotaxis, excess LDL cholesterol uptake, and release of pro-inflammatory cytokines. The dysregulated actions of these factors contribute to coronary atherosclerosis and restenosis [1].

IGF-I is a polypeptide hormone produced mainly by the liver in response to the endocrine GH stimulus, but it is also secreted by multiple tissues for autocrine/paracrine purposes. IGF1 has an important role in the development, cell differentiation, plasticity, and survival of the nervous system [2]. The bioavailability of IGF1 is regulated by its binding to IGF binding proteins (IGFBPs). Insulin-like peptides participate in neuroprotection and may have an important role in the pathophysiology of several neurologic disorders and as potential therapeutic targets for these conditions.

IGF-I exerts neuroprotective effects in both white and gray matter under different detrimental conditions. It is a key regulator of cell proliferation and an inhibitor of cell apoptosis and necrosis [3]. In the last decade, numerous studies have investigated the effect of IGF-I concentration on aging and different aging-related diseases, *e.g.*, cardiovascular disease (CVD) and cancer [4]. In population-based studies, high-normal levels of IGF-I have been reported to be associated with a moderately increased risk of several common cancers [5] and Parkinson's disease [6]. Low-normal IGF-I levels have been shown to be associated with the development of ischemic heart disease [7], congestive heart failure [8], diabetes among young subjects [9], frailty [10], acute aneurysmal subarachnoid hemorrhage [11], and Alzheimer's disease in men [12]. Roubenoff et al. [13] suggested that a decrease in the IGF-I level is a risk factor for mortality in the elderly. Low-normal levels of IGF-I is associated with increased mortality in ischemic heart disease and stroke [14].

Several epidemiologic studies have reported an inverse relation between plasma IGF-I levels and risk of ischemic stroke [15]–[16]. Serum IGF-I levels decline with increasing age, with lack of exercise, and in subjects with the metabolic syndrome [17]. Even after correcting for such confounders, a low serum IGF-I level is still associated with an increased risk of stroke [15]. However, because the etiology and pathogenesis of stroke are complex and multifactorial, it remains to be established whether the relation is causative. Thus, we sought to investigate the significance of serum IGF-I levels in a cohort of Chinese patients with acute ischemic stroke and to compare these levels with those of a control group.

## Subjects and Methods

All consecutive patients with first-ever acute ischemic stroke from August 1, 2011 to July 31, 2013 were recruited to participate in the study. Patients were defined according to the World Health Organization criteria [18] and had symptom onset within 24 hours. We excluded patients with malignant tumor, intracerebral hemorrhage, renal insufficiency, severe edema, febrile disorders, systemic infections, history of recent surgery or trauma during the preceding 2 months, autoimmune diseases and presence of diverse medical illness or current medications that influence serum IGF-I levels, and incomplete workups for cerebrovascular status.

Demographic and clinical data, including gender, age, and history of conventional vascular risk factors (hypertension, diabetes mellitus, atrial fibrillation, hyperlipoproteinemia, smoking habit, and alcohol abuse), were obtained. A neurologist assessed the stroke severity on admission by using the National Institutes of Health Stroke Scale (NIHSS; the NIHSS scores range from 0 to 34, with higher values reflecting more severe neurologic damage) [19]. The stroke subtype was classified according to the TOAST (Trial of Org 10172 in Acute Stroke Treatment) criteria [20], which distinguished large-artery arteriosclerosis, small-artery occlusion, cardioembolism, other causative factors, and undetermined causative factors. The clinical stroke syndrome was determined by applying the criteria of the Oxfordshire Community Stroke Project: total anterior circulation syndrome (TACS), partial anterior circulation syndrome (PACS), lacunar syndrome (LACS), and posterior circulation syndrome (POCS) [21]. Brain imaging (either CT or MRI) was done routinely within 24 hours after admission. MRI with diffusion-weighted imaging (DWI) was available for some patients. In those patients, DWI lesion volumes were determined by an experienced neurologist who was unaware of the clinical and laboratory results. The infarct volume was calculated by using the formula 0.5×a×b×c (where a is the maximal longitudinal diameter, b is the maximal transverse diameter perpendicular to a, and c is the number of 10-mm slices containing infarct) [22]–[23].

One hundred healthy people matched for age and gender were assigned to the normal group. Two hundred people matched for age, gender, and conventional vascular risk factors were assigned to the control group. A neurologist (not an author) reviewed the records of potential members of the normal and control groups to exclude the presence of stroke and other types of cerebrovascular disease. The median age in the normal group was 66 (IQR, 56–77) years, and 36% were women. This study was approved by the Institutional Review Board of The First Affiliated Hospital of Dalian Medical University. All participants were informed of the study protocol and gave their written informed consent according to the Declaration of Helsinki.

All blood samples were collected in fasting state on the first day of admission, and IGF-I levels were measured in accordance with standard detection methods in the biochemistry department of the hospital (Immulite 2000, Diagnostic Products Corp., Los Angeles, CA). Tests for routine serum biomarkers were done by standard detection methods. In our study, the lower detection limit for IGF-I was 25 ng/mL, and the detection range was 25–1600 ng/mL. The intra- and inter-assay coefficients of variation [CV] were 1.0–2.2% and 1.5%–2.4%, respectively. The median IGF-I level in the 100 healthy individuals was 158 ng/mL, which is slightly lower than that in the other population (172 ng/mL [12]).

The results were expressed as percentages for categorical variables and as medians (interquartile ranges,IQRs) for continuous variables. The Mann-Whitney U test and chi-square test were used to compare the two groups. Correlations among laboratory parameters were analyzed by using Spearman's rank correlation test. Associations between the severity of stroke evaluated by NIHSS scores and the serum levels of IGF-I were assessed by using ordered logistic regression models with multivariate adjustment for possible confounders, for instance, age, gender, alcohol abuse, smoking habit, hypertension, diabetes, atrial fibrillation, hyperlipoproteinemia, infarct volume, and serum levels of white blood cells, triglyceride, cholesterol, high-density lipoprotein (HDL), low-density lipoprotein (LDL), D-dimer, glucose, high-sensitivity C-reactive protein (hs-CRP), and homocysteine (HCY). Logistic regression analysis was used to evaluate the risk of stroke according to serum IGF-I levels, after adjustment for the above possible confounders and NIHSS scores. The results were expressed as adjusted OR (odds ratios), with the corresponding 95% confidence interval (CI). Receiver operating characteristic (ROC) curves were used to evaluate the accuracy of serum IGF-I in predicting AIS. The area under the curve (AUC) was calculated as a measure of the accuracy of the test. All statistical analyses were done with SPSS for Windows, version 20.0 (SPSS Inc., Chicago, IL, USA). Statistical significance was set at p<0.05.

## Results

A total of 221 patients with first-ever AIS were included in this study. Table 1 shows the baseline characteristics of these patients, of which 141 (63.8%) were males. The median age was 66 years (IQR, 57–77). The median NIHSS score on admission was 7 points (IQR, 3 to 12). The median time from symptom recognition to hospital admission was 7.3 hours (IQR 4.4–13.7), and 152 patients (68.8%) were admitted within 12 hours of symptom recognition.

**Table 1:** Baseline characteristics of acute ischemic stroke patients and control cases.

Characteristics	Patients (n = 240)	Control cases (n = 200)	Normal cases (n = 100)
Age (years), median(IQR)	66(57–77)	66(56–77)	66(56–77)
Male sex (%)	141(63.8)	128(64.0)	64(64.0)
Infarct volume(mL, IQR; n = 168)	10(7–22)	-	-
Stroke severity, median NIHSS score (IQR)	7(3–12)	-	-
The time from symptom to admission (hours), median(IQR)	7.2(4.4–13.7)	-	-
Vascular risk factors no. (%)			
Hypertension	158(71.5)	144(72.0)	-
Diabetes mellitus	62(28.1)	56(28.0)	-
Atrial fibrillation	49(22.2)	45(22.5)	-
Coronary heart disease	53(24.0)	48(24.0)	-
Hypercholesterolemia	65(29.4)	60(30.0)	-
Family history for stroke	52(23.5)	44(22.0)	12(12.0)
Alcohol abuse	48(21.7)	44(22.0)	11(11.0)
Smoking habit	45(20.4)	40(20.0)	15(15.0)
Clinical findings median(IQR)			
Temperature (°C)	37.0(36.5–37.5)	36.5(36.2–36.8)	36.4(36.2–36.7)
Heart rate (beats min^−1^)	83(72–91)	81(69–88)	80(71–86)
BMI (kg m^−2^)	23.9(22.6–26.8)	24.2(23.1–27.1)	23.8(22.4–26.4)
Systolic blood pressure(mmHg)	156(144–175)	152(142–173)	130(125–136)
Diastolic blood pressure(mmHg)	95(84–99)	93(82–97)	84(79–88)
Laboratory findings (median, IQR)			
Leucocyte count (×10^3^ m L^−1^)	8.3(6.5–9.6)	8.2(6.4–9.5)	7.8(7.2–8.7)
Glucose(mmol L^−1^)	6.03(5.66–6.54)	5.99(5.52–6.59)	5.44(5.25–5.86)
Hs-CRP(mgL^−1^)	0.57(0.35–0.98)	0.41(0.27–0.68)	0.25(0.14–0.33)
D-dimer(mg L^−1^)	0.78(0.32–2.03)	0.49(0.21–1.13)	0.32(0.21–0.53)
Stroke syndrome no. (%)			
TACS	28(11.7)	-	-
PACS	89(40.3)	-	-
LACS	46(20.8)		
POCS	58(26.2)	-	-
Stroke etiology no. (%)			
Small-vessel occlusive	45(20.4)	-	-
Large-vessel occlusive	44(19.9)		
Cardioembolic	90(40.7)	-	-
Other	20(9.0)	-	-
Unknown	22(10.0)	-	-

IQR, interquartile range; TACS, total anterior circulation syndrome; LACS, lacunar syndrome; PACS, partial anterior circulation syndrome; POCS, posterior circulation syndrome; NIHSS, National Institutes of Health Stroke Scale; Hs-CRP, high sensitivity C-reactive protein.

The median serum IGF-I levels were significantly (P = 0.011) lower in the AIS patients compared to control cases (129; IQR, 109–153 ng/mL and 140; IQR, 125–159 ng/mL, respectively; Figure 1). Similarly, the median serum IGF-I levels were also significantly (P = 0.000) lower compared to normal cases (129; IQR, 109–153 ng/mL and 158; IQR, 137–173 ng/mL, respectively; Figure 1). There was a modest correlation between serum IGF-I levels and age (r = −0.200, P = 0.004), as shown in Fig. 2a, and inverse correlations between the levels of IGF-I and the NIHSS (r = −0.453, P = 0.000; Fig. 2b) and Hs-CRP levels (r = −0.178, P = 0.009; Fig. 2c). A significant positive trend between serum IGF-I levels and NIHSS score (P = 0.006) was observed in the ordered logistic regression even after multivariate adjustment for the above-mentioned possible confounders.

**Figure 1:** Serum IGF-I levels in acute ischemic stroke patients, control and normal group. Mann–Whitney U-test. All data are medians and in-terquartile ranges (IQR). Significantly higher in stroke patients as compared to control cases (p = 0.011); Significantly higher in stroke patients as compared to normal cases (p = 0.000).

**Figure 2:** Correlation between serum IGF-I levels and others predictors. (a) Correlation between serum IGF-I levels and age; (b) Correlation between the serum IGF-I levels and the National Institutes of Health Stroke Scale (NIHSS) score; (c) Correlation between serum IGF-I levels and Hs-CRP; (d) Correlation between serum IGF-I levels and infract volume.

In this study, MRI data were available for 178 patients, and there was a negative correlation between the serum levels of IGF-I and the infarct volume (r = −0.263, P = 0.000; Fig. 2d). A significant inverse trend between serum IGF-I levels and infarct volume (P = 0.012) persisted even after adjustment for the above covariates. In addition, there were no significant correlations between serum levels of IGF-I and other variables, namely, sex, stroke syndrome, stroke etiology, glucose, and HCY (P>0.05).

In the model matching for gender and age, the optimal cutoff value for serum IGF-I levels as an indicator of an auxiliary diagnosis of AIS was projected to be 135 ng/mL, which yielded a sensitivity of 77.8% and a specificity of 72.4%, with the area under the curve at 0.787 (95% CI: 0.694–0.848). In the univariate model matching for gender and age, IGF-I as a continuous variable was associated with an increased risk of AIS (OR: 1.003, 95% CI: 1.001–1.008; *P* = 0.009). Further, we found that an increased risk of AIS was associated with IGF-I levels ≤135 ng/mL (unadjusted OR: 4.17, 95% CI: 2.52–6.89; *P* = 0.000). This relationship was confirmed in the dose-response model. In the multivariate analysis, an increased risk of AIS was still associated with IGF-I levels ≤135 ng/mL (OR: 2.16, 95% CI:1.33–3.52; P = 0.002) after adjusting for possible confounders.

## Discussions

In our study, we reported that serum IGF-I levels were significantly reduced in cases of first AIS compared with control cases. For the entire group, after adjusting for other possible risk factors, a reduced IGF-I level was an independent risk factor for stroke, and serum IGF-I levels ≤135 ng/mL were associated with a 2.16-fold increase in AIS. Furthermore, we found that serum IGF-I levels dropped with increasing severity of stroke as defined by the NIHSS score, and there were inverse correlations that linked the levels of IGF-I to the Hs-CRP levels and the infarct volume.

In the present study, no difference in IGF-I levels was observed between genders. Many other studies also failed to show a distinction between genders [24]–[25]. Roubenoff et al [13] reported that serum IGF-I levels decreased with age in a community dwelling populations, which was supported by our findings. In addition, selvamani et al. [14] reported that stroke severity in older females rat were associated with decreased IGF-I, which was also consistent with our results. On the contrary, the baseline stroke severity did not differ between high- and low-IGF-I groups in one study [26]. We found an inverse correlation between the levels of IGF-I and the infarct volume. Previous studies indicated that systemic administration of IGF-I injection results in decreased infarct volume [27]–[28].

Whether higher levels of circulating IGF-I are an accelerator or a consequence of AIS remains uncertain. First, accumulating evidence has suggested that insufficient IGF-I levels play a role in vascular diseases, such as atherosclerosis and restenosis [29]. Interestingly, atherosclerotic plaque involves many factors, and IGFs play a relevant role. Type I IGF receptors are present on smooth muscle cells, inflammatory cells, and arterial endothelial cells within the atherosclerotic lesion [1]. Second, several in vitro studies have shown that IGF-I induces cell cycle changes resulting in VSMC proliferation and migration. VSMC apoptosis occurs in the evolutionary process of atherosclerotic plaques [30]. It is likely that macrophage-derived IGF enhances cellular LDL uptake and degradation, as well as the macrophage cholesterol esterification rate [31]. Third, atherosclerosis is characterized by a chronic low-grade inflammatory state 32]. Recent studies have suggested that IGF-I exerts anti-inflammatory properties by decreasing the expression of pro-inflammatory cytokines [33]. Conversely, Roubenoff et al. [13] found a relationship between serum IGF-I and serum interleukin 6 [34]. In our study, we also found an inverse correlation between the levels of IGF-I and of Hs-CRP. Interestingly, the protective effect of IGF-I was found to be independent of inflammatory markers, either systemic (CRP and fibrinogen) or local (ICAM-1) [32]. This suggests that the major effects of IGF-I are independent of inflammation control. Fourth, IGF-I plays a main role in restoring mitochondrial dysfunction during aging by increasing mitochondrial membrane potential, reducing oxygen consumption, and increasing ATP synthesis, which in turn minimize the cytochrome release to the cytoplasm and subsequently promote neural survival by decreasing caspase-induced apoptosis [35]. Azzouzi et al. [36] confirmed the role of the IGF-I signaling pathway in the protection of cardiomyocytes under ischemic and hemodynamic loading conditions. Impaired IGF-I signaling has already been linked to increased oxidative stress and mitochondrial dysfunction in neuronal cells [37]. Fifth, a number of studies have shown the importance of IGF-I in many processes of immune function [38]. IGF-I plays important roles in T lymphocyte development and function. Specifically, it can increase the number of CD4+CD8+ immature T cells in rat thymus and spleen and promotes T cell survival [35]. IGF-I has been reported to enhance IL-7-dependent B-cell proliferation in parallel with the c-kit ligand, as well as to potentiate IL-7 promotion of pro-B-cell expansion [35]. Lastly, IGF-I penetrates into the brain and could potentially provide fast and efficient treatment to prevent chronic effects of stroke [39]. IGF-I protects neurons against excitotoxicity and oxidative stress, as indicated by in vitro experiments showing that IGF-I inhibits glutamate-, nitric oxide-, and hydrogen peroxide-induced apoptosis [26]–[27]. IGF-I also protects oligodendrocyte precursors from cytotoxicity [40]. In addition to having protective effects, IGF-I can also influence recovery from ischemic stroke through regeneration [27]. Furthermore, it is able to modulate brain plasticity by influencing neurite outgrowth, synaptogenesis, neuronal excitability, and neurotransmitter release [41].

Some limitations of this observational study merit consideration. First, serum IGF-I levels were measured only once after stroke onset; additional measurements in the days thereafter would have been of interest. Second, follow-up data are lacking. In ischemic stroke, low IGF-I concentrations may predict poor outcome in humans [42]–[43]. Further studies are needed to determine whether serum IGF-I levels predict outcomes after a stroke in our population. Furthermore, the biological effects and bioavailability of IGF-I are modulated through IGFBPs, which control IGF-I access to cell surface receptors. Unfortunately, we did not have IGFBPs; therefore, our results do not fully represent biologically active IGF-I. Finally, IGF-I measurements were done after the stroke and thus may not accurately reflect pre-stroke exposure.

In conclusion, lower IGF-I levels (≤135 ng/mL) are significantly related to risk of stroke, independent from other traditional and emerging risk factors, suggesting that they may play a role in the pathogenesis of AIS. Thus, IGF-I levels should be considered as a routine risk factor for stroke in the Chinese population, and further post-ischemic IGF-I therapy may be beneficial for stroke. We suggest routing screening of serum IGF-I levels to prevent stroke in the Chinese population. However, before a broad implementation of this recommendation, additional studies are needed for external validation.
